# Violations of Personal Space by Individuals with Autism Spectrum Disorder

**DOI:** 10.1371/journal.pone.0103369

**Published:** 2014-08-06

**Authors:** Daniel P. Kennedy, Ralph Adolphs

**Affiliations:** 1 Department of Psychological and Brain Sciences, Indiana University, Bloomington, Indiana, United States of America; 2 Division of Humanities and Social Sciences, California Institute of Technology, Pasadena, California, United States of America; 3 Division of Biology, California Institute of Technology, Pasadena, California, United States of America; Ecole Normale Supérieure, France

## Abstract

The ability to maintain an appropriate physical distance (i.e., interpersonal distance) from others is a critical aspect of social interaction and contributes importantly to real-life social functioning. In Study 1, using parent-report data that had been acquired on a large number of individuals (ages 4–18 years) for the Autism Genetic Resource Exchange and the Simons Simplex Collection, we found that those with Autism Spectrum Disorder (ASD; n = 766) more often violated the space of others compared to their unaffected siblings (n = 766). This abnormality held equally across ASD diagnostic categories, and correlated with clinical measures of communication and social functioning. In Study 2, laboratory experiments in a sample of high-functioning adults with ASD demonstrated an altered relationship between interpersonal distance and personal space, and documented a complete absence of personal space in 3 individuals with ASD. Furthermore, anecdotal self-report from several participants confirmed that violations of social distancing conventions continue to occur in real-world interactions through adulthood. We suggest that atypical social distancing behavior offers a practical and sensitive measure of social dysfunction in ASD, and one whose psychological and neurological substrates should be further investigated.

## Introduction

Social dysfunction is one of the key diagnostic criteria in Autism Spectrum Disorder (ASD), and is often the single most disabling component for individuals with an ASD who otherwise might be considered high functioning. Research into the cognitive and neurobiological basis of social dysfunction has focused to a large extent on a few particular domains of social processing-most notably, face processing and mentalizing abilities [1]–[3]. Comparatively neglected has been research on other important aspects of social functioning, especially as they relate to real-world social interactions that can often be difficult to quantify. One such behavior is the regulation of social (i.e., interpersonal) distance, or the physical distance maintained between individuals during social interaction [4]. Though seemingly automatic and effortless, one’s determination of the appropriate distance from others is a complex and dynamic social judgment that is simultaneously dependent on a number of factors, including person familiarity, cultural norms, emotional state, age, gender, and situational context, along with other variables. Social distance regulation is critical for successful social interaction, as its dysregulation can lead to personal space violations (and ensuing feelings of discomfort), as well as the inadvertent miscommunication of social intentions (e.g., aggression, defensiveness, social interest or disinterest, etc.) [4].

Anecdotally, parents, teachers, and clinicians have all described a lack of awareness of social distance norms in individuals with ASD [5], yet support for these claims is still somewhat limited. Several studies have found abnormalities in social distancing in ASD [6]–[11], but these studies generally used smaller sample sizes, did not apply modern research criteria for an ASD diagnosis, and/or did not test a well-matched comparison sample, thus highlighting the need for further studies. One very recent exception to this found larger-than-normal interpersonal distance preferences in children with ASD, and that interpersonal distance failed to modulate as a function of social familiarity in this group [12]. Other studies using virtual reality have demonstrated that adolescents with an ASD seem to not respect the space of virtual characters [13], including walking directly in-between two characters seemingly engaged in a conversation with one another. However, it is currently unknown whether these types social distancing violations measured using virtual reality generalize to social distancing in the real world. In addition, these earlier studies focused solely on quantifying interpersonal distance – i.e., the readily observable physical distance between people. Less understood is whether or not individuals with ASD have an altered sense of personal space (i.e., the physical space around someone into which intrusion causes discomfort), and if so, whether this alteration relates to abnormal interpersonal distance preference.

In the current study, we took two complementary approaches to investigating the regulation of social distance in ASD – questionnaire-based data on a large number of individuals with ASD and their unaffected siblings (Study 1) and more tightly controlled laboratory experiments using the stop-distance technique [14] (Study 2). In Study 1, we analyzed phenotypic data from two large databases, the Simons Simplex Collection (SSC) and the Autism Genetic Resource Exchange (AGRE). We focused our analysis on data from the Social Responsiveness Scale (SRS), a 65-item parent- or teacher-report questionnaire designed to quantify the severity of autistic symptoms [15]. One item on the SRS explicitly assesses social distance violations at close proximity (Item 55), and we used this item as a starting point for our analyses. Our specific goals were as follows: (a) to compare probands (i.e., affected individuals; in this case, individuals with autism) and their siblings on social distance regulation, and (b) to determine the relationship between social distancing and various other parent-reported behaviors and clinical measures. In Study 2, we used controlled laboratory experiments with high-functioning adults with ASD and matched controls to complement and extend the above questionnaire-based approach. Specifically, we sought to (c) further explore whether and how such abnormalities may manifest in adulthood, and (d) attempt to gain preliminary insight into the possible psychological mechanisms underlying these social distance abnormalities. Together, such results would quantify the prevalence of social distance abnormalities in autism, identify behaviors and domains of functioning that co-segregate with this measure, and possibly suggest potential subtypes of autism (i.e., those with interpersonal distance abnormalities and those without) that may ultimately be traceable to distinct neurological and genetic profiles.

## Methods

### Study 1

#### Datasets

Phenotypic data were acquired from two publicly available databases: AGRE and SSC. The use of these de-identified data was approved by the Institutional Review Board at the California Institute of Technology. The principal difference between the two datasets was that the AGRE sample included only multiplex families (i.e., 2 or more affected individuals (in this case, children) within the family), whereas the SSC included only simplex families (i.e., only 1 affected individual). For the AGRE sample, we only included individuals that met AGRE designations of autism, which were based on fully meeting cutoff criteria on the Autism Diagnostic Interview – Revised (ADI-R) [16]. Individuals with AGRE designations of “Not Quite Autism” or “Broad Spectrum”, given to those individuals that did not fully meet ADI-R cutoffs, were excluded from all analyses due to their ambiguous diagnostic status. Furthermore, since the ADI-R alone cannot differentiate between ASD subtypes, this dataset was not included in any analysis involving diagnostic subtypes. SSC diagnoses were based on the ADI-R, the Autism Diagnostic Observation Schedule (ADOS) [17], and expert clinical judgment, providing diagnoses of Autistic Disorder, Asperger’s Syndrome, or PDD-NOS (Pervasive Developmental Disorder - Not Otherwise Specified).

For our analyses of both the AGRE and SSC datasets, a single ASD proband was matched with a single unaffected sibling from the same family (ASD-sib pairs). For all pairs, when multiple ASD proband or sibling options were available, individuals were chosen to best match first on gender, and then on age. Before pairs were created, specific exclusionary criteria were first applied to all cases, as detailed in Table 1 (AGRE) and Table 2 (SSC). This consisted of the following exclusionary criteria: 1) too many missing responses (greater than 6 SRS items), 2) SRS data acquired from invalid respondents (i.e., non-parent or caregiver), 3) younger than 4 years or older than 18 years, 4) evidence for non-ideopathic autism (i.e., cases with a specifically known cause, such as identified chromosomal abnormalities like Fragile X Syndrome), 5) did not meet diagnostic criteria for an ASD, 6) unaffected siblings with total SRS scores greater than T-Score cutoffs for clinically significant social impairment (potentially indicative of an undiagnosed ASD), 7) 1 individual from monozygotic twins, or 2 individuals from monozygotic triplets, and 8) families that did not meet the multiplex designation in the AGRE sample (i.e., only 1 ASD proband) or had only 1 child in the SSC sample. The final sample consisted of 82 ASD-sib pairs (164 individuals) from the AGRE dataset (Table 1) and 684 ASD-sib pairs (1368 individuals) from the SSC dataset (Table 2). In the SSC dataset, the ASD group was comprised of 467 individuals with autism, 81 with Asperger’s Syndrome, and 136 with a PDD-NOS diagnosis. Thus, after applying our exclusionary criteria, our final sample included 1532 individuals in total, consisting of 766 ASD individuals and 766 of their siblings (see **Table 3** for a detailed characterization of these groups).

**Table 1:** A list of the exclusionary criteria applied to AGRE dataset.

AGRE Subject Selection	
# of Records	Exclusion Criteria
1593	Parent-Report SRS
1172	No record in pedigree
1152	Invalid respondent or missing too many responses
1097	Age less than 4 years or greater than 18 years
1065	non-ideopathic autism
825	probands did not meet ADI-R criteria for Autistic Disorder
804	unaffected siblings with total SRS scores greater than published T-scorecutoffs (indicative of a potentially undiagnosed ASD)
801	duplicate entries
788	if monozygotic twins, triplets, etc., removed all except 1
623	removed simplex families
**82**	**Total ASD-Sib Pairs**

**Table 2:** A list of the exclusionary criteria applied to SSC dataset.

SSC Subject Selection	
# of Records	Exclusion Criteria
1825	Parent-Report SRS
1825	No record in pedigree
1824	duplicate entries
1816	non-simplex families
1816	Invalid respondent or missing too many responses
1800	Age less than 4 years or greater than 18 years
1745	non-ideopathic autism
1745	probands did not meet best-estimate diagnosis of ASD
1713	unaffected siblings with total SRS scores greater than published T-scorecutoffs (indicative of a potentially undiagnosed ASD)
1700	if monozygotic twins, triplets, etc., removed all except 1
1474	remove families with only 1 child
**684**	**Total ASD-Sib Pairs**

**Table 3:** Subject characteristics for each group.

Subject Characteristics			
		ASD	Siblings
**Mean Age (±SD)**		114.7 (±42.6) months	112.7 (±38.9) months
**Male:Female ratio**		5.03∶1.0	0.87∶1.0
**Vineland**		73.3 (±13.3)	104.7 (±11.6)*
**Total SRS score**		102.6 (±28.9)	17.5 (±11.7)
**ADI-R**	*Social*	20.7 (±5.8)	-
	*Verbal Comm*	16.7 (±4.2)	-
	*Non-verbal Comm*	9.3 (±3.5)	-
	*RSB*	6.4 (±2.6)	-

* = derived from the SSC dataset alone, since this information was not acquired from siblings in the AGRE dataset.

RSB = restricted, repetitive, and stereotyped patterns of behavior; SD = standard deviation.

#### Social Responsiveness Scale

The SRS is a 65-item parent- or teacher-report questionnaire that quantifies the severity of autistic impairment [15]. While designed to measure social deficits on a continuum, it has also demonstrated diagnostic utility [18]. For the present analyses, due to the larger number of parent-report compared to teacher-report data available, we restricted our analysis to parent-report data only. Individual SRS items are rated on a 4-point scale (from 0 to 3), with higher scores reflecting a higher frequency of autistic-like behaviors. Item 55 deals explicitly with social distancing (i.e., “knows when he or she is too close to someone or is invading someone’s space”). Two additional items on the SRS were also of interest as they relate to the construct of social distance regulation - item 63: “Touches others in an unusual way (e.g., he or she may touch someone just to make contact and then walk away without saying anything)”, and item 56: “Walks in between two people who are talking”. We examined these items, as well as a third that turned out to be highly correlated with item 55 (item 52; “Knows when he or she is talking too loud or making too much noise”).

Because the single item ratings are ordinal data, we used non-parametric tests for all analyses, unless stated otherwise. Furthermore, because the distributions of scores on item 55 did not differ between AGRE and SSC datasets (U = 123535.5, Z = −0.42, p = 0.67, n_1_ = 164, n_2_ = 1368, Mann-Whitney U test), these datasets were combined for all analyses, unless stated otherwise. Based on previous studies, anecdotal reports, and our own experiences, we hypothesized that individuals with an ASD would be more likely to exhibit social distancing abnormalities, compared to their unaffected siblings. All statistical tests were two-tailed. In addition, all significant correlations reported below survive Bonferroni correction for multiple comparisons.

### Study 2

#### Participants

18 ASD participants and 20 control participants took part in this study. Diagnosis of an ASD was confirmed using the ADOS (all module 4), ADI-R or SCQ (when a parent or guardian was available), and expert clinical judgment according to DSM-IV criteria. Groups did not differ on age, gender, or verbal, performance, or full-scale IQ (all p>0.3) (Table 4). This experiment was approved by Caltech’s Institutional Review Board (IRB), and all participants gave written informed consent.

**Table 4:** Participant characteristics for Study 2.

Subject Characteristics			
		ASD (n = 18)	Controls (n = 20)
**Mean Age (±SD)**		27.1 (±7.7) years	26.8 (±4.2) months
**Males/Females**		13/5	16/4
**Total SRS score**		98.1 (±28.2)*	-
**WASI**	*Verbal*	111.7 (±17.4)	113.7 (±8.3)
	*Performance*	108.2 (±9.7)	108.6 (±9.0)
	*Full Scale*	110.4 (±12.3)	112.6 (±8.1)
**ADOS**	*Comm*	4.5 (±1.5)	-
	*Social*	9.0 (±3.9)	-
	*Repetitive*	1.6 (±1.4)	-

* = SRS scores were not available from controls, and unavailable for 3 of the ASD participants.

#### Task

In the first half of the experiment (Interpersonal Distance Condition), participants were instructed to approach the experimenter and stop at the location that felt perfectly comfortable to them. They started from approximately 3 meters away, and always approached the same experimenter, who maintained a consistent neutral expression and tried to maintain equal amounts of eye contact across participants. Once they chose the location that felt most comfortable, participants were asked to hold still while chin-to-chin distance was measured using a digital laser distance measurer (Bosch, model DLR165K). Distances were measured twice in immediate succession, and averaged together to account for slight variations due to body sway.

In the second half of the experiment (Personal Space Condition), the same procedures were carried out, but this time participants were asked to stop at the location that just started to feel uncomfortable to them. In addition, participants were instructed that if there was no point at which they felt uncomfortable, then they should walk as close as possible to the experimenter without physically touching them, and then to verbally tell the experimenter so. Participants completed 4 trials of each type, with the 4 Interpersonal Distance trials always preceding the 4 Personal Space trials. The order of conditions was fixed to avoid the concern that the discomfort experienced by participants during the Personal Space trials would influence their Interpersonal Distance judgments.

After all the trials were completed, participants were asked to verify that they understood the instructions by verbally explaining to the experimenter why they stopped where they did on the various trials. All participants demonstrated full understanding of the instructions (i.e., stopping at a comfortable distance for Interpersonal Distance trials, and stopping at a distance where they started to feel slightly uncomfortable for Personal Space trials), as would be expected in this group of high-functioning ASD adults and age-, gender-, and IQ-matched controls.

The relationship between mean Interpersonal Distance and mean Personal Space were examined using regression analyses, and the residuals of the regression were compared across groups.

## Results

### Study 1

After applying exclusionary criteria, there were no differences between groups in terms of age (proband mean (±SD) = 112.7 months (±38.9); sibling = 114.7 months (±42.6); t(1530) = 0.96, p = 0.34, independent samples t-test). Not surprisingly, groups did differ in terms of total SRS scores (probands = 99.6 (±27.3); siblings = 17.8 (±11.8); t(1530) = 76.2, p<0.0001) and Vineland standard composite scores (probands = 73.3 (±13.3); siblings = 104.7 (±11.6); t(1403) = 46.9, p<0.0001) (Table 3).

#### Social Distancing

As hypothesized, there was a difference between probands and siblings on social distancing (item 55), with ASD probands (mean = 2.22, SD = 0.94) rated as less aware of being too close and more prone to personal space invasions than their unaffected siblings (mean = 0.70, SD = 0.95; U = 789911.5, Z = −24.32, p<0.0001, n_1_ = n_2_ = 766, Mann-Whitney U test; **Figure 1a**). This was true for both the AGRE dataset (ASD mean = 2.38 (0.90), sibling mean = 0.46 (0.77), U = 9561, Z = −9.63, p<0.0001, n_1_ = n_2_ = 82) and the SSC dataset (ASD mean = 2.20 (0.95), sibling mean = 0.73 (0.97); U = 625713, Z = −22.37, p<0.0001, n_1_ = n_2_ = 684), when analyzed separately. The difference in scores between ASD-sibling pairs was slightly larger in the AGRE sample compared to the SSC sample (t(764) = 2.96, p = 0.003, independent samples t-test). Furthermore, ASD and sibling groups remained different even when including those siblings with elevated total SRS scores (AGRE: ASD mean = 2.40 (0.85), sibling mean = 0.53 (0.81), U = 11262, Z = −10.01, p<0.0001, n_1_ = n_2_ = 89; SSC: ASD mean = 2.20 (0.76), sibling mean = 0.76 (0.98), U = 658433.5, Z = −22.33, p<0.0001, n_1_ = n_2_ = 703). Examination of the frequency histograms for each group reveals how well this single item (item 55) differentiates probands from their siblings (see **Figure 1b**). 78.6% of ASD-sib pairs had higher scores for probands than siblings, while the converse was true only 6.5% of the time (scores were equal for the remaining 14.9%). Relative to all other items on the SRS, this item ranks 21st out of 65 items in terms of differentiating groups (i.e., it is better than roughly two-thirds of all SRS items). There were no differences in mean ratings on this measure across the various ASD sub-categories (provided in the SSC dataset; autism mean (SD) = 2.20 (0.94); Asperger’s mean = 2.22 (0.99); PDD-NOS mean = 2.17 (0.94); H(2) = 0.47, p = 0.79, n_1_ = 467, n_2_ = 81, n_3_ = 136, Kruskal-Wallis test).

**Figure 1:** Ratings on item 55 (awareness of social distancing) in ASD and siblings. A) Mean ratings for each group; error bars reflect standard error of the mean (SEM). B) histograms showing the number of individuals who received each rating on item 55. Scores range from 0 to 3, with higher scores reflecting a greater frequency of social distancing abnormalities.

Ratings on item 55 correlated with total SRS scores, after removing the contribution of item 55 to the total SRS score (probands: r = 0.29, p<0.0001, siblings: r = 0.42, p<0.0001; Spearman correlation). ASD probands with higher scores on item 55 (ratings of 2 or 3) had higher total SRS scores (after removing the contribution of item 55; mean = 100.1 (25.9) out of a possible 195) compared to ASD probands with lower scores on this item (ratings of 0 or 1; mean = 86.6 (28.5); U = 47321, Z = −5.21, p<0.0001, n_1_ = 609, n_2_ = 157, Mann-Whitney U test). Given that scores on SRS items are generally positively correlated with one another [19], (in the present ASD sample, mean correlation across all pairwise item correlations, r = 0.19, SD = 0.10), it is not surprising that those with high scores on item 55 have higher overall scores. Interestingly, however, the three SRS items with the highest correlations to item 55 all seem to relate to social distancing and personal space: item 52 (r = 0.42, p<0.0001): “Knows when he or she is talking too loud or making too much noise”; item 63 (r = 0.31, p<0.0001): “Touches others in an unusual way (e.g., he or she may touch someone just to make contact and then walk away without saying anything)”; and item 56 (r = 0.30, p<0.0001): “Walks in between two people who are talking” (see **Figure 2**). Correlations between item 55 and these items remained the three strongest even after accounting for age (partial correlations: r = 0.42, r = 0.31, r = 0.30, respectively; all p<0.0001) and Vineland scores (partial correlations: r = 0.39, r = 0.28, r = 0.27, respectively; all p<0.0001).

**Figure 2:** Correlations between ratings on item 55 (white) and all other SRS items. The three items with the highest correlations were items 52 (“Knows when he or she is talking too loud or making too much noise”), 56 (“Walks in between two people who are talking”), and 63 (“Touches others in an unusual way (e.g., he or she may touch someone just to make contact and then walk away without saying anything)”), all of which relate to the concept of social distancing.

#### Correlations with ADI-R

There were positive correlations between item 55 and the ADI-R social subscale (r = 0.13, p = 0.0004) and ADI-R communication subscale (verbal: r = 0.11, p = 0.006; non-verbal: r = 0.13, p = 0.0005), but not with the ADI-R restricted and stereotyped behaviors (RSB) subscale (r = −0.002, p = 0.96). The pattern of results remained after controlling for age (social, verbal communication, and non-verbal communication, r = 0.16, r = 0.12, r = 0.15, respectively, all p<.002; RSB, r = 0.004, p = 0.90, non-parametric partial correlation), but not after controlling for Vineland standard composite scores (all r<0.06, all p>0.13).

#### Effects of age, gender and adaptive functioning

The above described results of differences between ASD probands and siblings on item 55 cannot simply be explained by age effects. While there were slight but significant correlations between item 55 and age in both the ASD and sibling groups (probands: r = −0.14, p<0.0001; siblings: r = −0.30, p<0.0001; Spearman correlation), groups were well-matched with respect to age. Furthermore, group differences were found at every age from 4 years to 18 years (see **Figure 3**; for all age bins, p<0.005, Mann-Whitney U test). Lastly, since the age of the control group was slightly lower than the ASD group, and since lower ages correspond to higher item 55 scores, one might, if anything, have expected to see higher scores in the sibling group compared to the ASD group if age were driving the results (i.e., an effect opposite to that observed). The results also could not be explained by differences in the number of males and females across proband and sibling groups (a consequence of the higher ratio of male:female individuals with an ASD), as there were no differences on item 55 ratings between male and female siblings (mean (SD) = 0.74 (0.98) and 0.67 (0.93), respectively; U = 139431.5, Z = 1.06, p = 0.29, n_1_ = 356, n_2_ = 410, Mann-Whitney U test), nor between male and female probands (2.24 (0.92) and 2.10 (1.04), respectively; U = 46262, Z = 1.17, p = 0.24, n_1_ = 639, n_2_ = 127, Mann-Whitney U test).

**Figure 3:** Ratings on item 55 (awareness of social distancing) in ASD and siblings across age bins (from 4 years to 18 years). Error bars reflect standard error of the mean (SEM). Group differences were present at every age bin (all p<0.005, Mann-Whitney U test).

Finally, we ran an additional analysis to ensure that differences in social distancing between groups could not be accounted for by group differences in adaptive functioning, as measured with the Vineland Adaptive Behavior Scales. This was of particular concern since there were group differences in Vineland composite scores (see above results and Table 3), and because item 55 was negatively correlated with Vineland scores in the autism group (r = −0.19, p<0.0001). Therefore, we created a subsample of the ASD and siblings groups that were well-matched on total Vineland scores, by selecting and comparing the lowest performing 20% of the sibling group and the highest performing 20% of the ASD group (ASD mean (SD) = 90.7 (5.4); Sibling mean (SD) = 90.0 (4.0); U = 21461, Z = −0.30, p = 0.76, n_1_ = n_2_ = 147, Mann-Whitney U test). Group differences on item 55 remained when using this subsample (ASD mean (SD) = 2.03 (0.95); Sibling mean (SD) = 0.82 (0.96); U = 28158, Z = 9.18, p<0.0001, n_1_ = n_2_ = 147, Mann-Whitney U test). Similarly, when we restricted our analysis to groups matched on the socialization score of the Vineland (ASD mean (SD) = 89.2 (6.16), Sibling mean (SD) = 88.4, (4.50)), groups remained different on item 55 (ASD mean (SD) = 1.96 (1.03); Sibling mean (SD) = 0.81 (0.97); U = 27702, Z = 8.55, p<0.0001, n_1_ = n_2_ = 147, Mann-Whitney U test).

### Study 2

Groups did not differ in terms of mean interpersonal distance (ASD = 79.9 (24.1); controls = 73.7 (17.6); [t(36) = 0.91, p = 0.37]) or mean personal space (ASD = 42.8 (29.5); controls = 42.8 (12.3); [t(36) = 0.002; p = 0.998]). Furthermore, both groups displayed a positive relationship between personal space and interpersonal distance preferences. This relationship was stronger in the control group (r = 0.881, p<0.0001) compared to the ASD group (r = 0.562, p 0.0152) (see **Figure 4a and 4b**).

**Figure 4:** Relationship between personal space and interpersonal distance preferences in ASD and control adults. The correlation between these two measures is stronger in the control group (Panel A; r = 0.881, p<0.000001) than in the ASD group (Panel B; r = 0.562, p = 0.0151). Residuals were derived from regression lines fit to each group separately. Absolute values of the residuals are plotted for control and ASD groups (Panel C). Groups were different on this measure (t(36) = 2.95, p = 0.0055), with the ASD group displaying greater residuals, indicating a less tight relationship between personal space and interpersonal distance preferences.

To quantify the difference in the degree to which personal space predicts interpersonal distance preference in the two groups, a regression line was fit for each group separately [ASD: *b* = 0.46; r^2^ = 0.316, F(1,16) = 7.4, p = 0.0151; Controls: *b* = 1.26; r^2^ = 0.776, F(1,18) = 62.4, p<0.000001]. Residuals for each individual subject were then derived from their respective regression lines, and the absolute value of the residuals were compared between groups, providing a measure of how much a particular individual deviates from the regression model. We found that the groups were different from one another (t(36) = 2.95, p = 0.0055), with the ASD group having higher residuals (mean±SD = 15.3±12.2) compared to the control group (6.5±4.9) (see **Figure 4c**), indicating a less tight relationship between personal space and interpersonal distance preferences in ASD. Close examination of **Figure 4b** also reveals that 3 individuals with ASD had no sense of personal space. Importantly, these group differences were not simply driven by these individuals, since the pattern of results were unchanged if these three individuals were first excluded from the analysis (new ASD regression: ASD: *b* = 0.61; r^2^ = 0.325, F(1,13) = 6.26, p = 0.026; ASD mean = 16.4±12.8; Control mean = 6.5±4.9; group difference: t(33) = 3.16, p = 0.0034). Furthermore, the results remained unchanged if a single regression line was calculated using data pooled across both groups together [*b* = 0.59; r^2^ = 0.38, F(1,36) = 22.2, p<0.0001; ASD mean = 16.5±11.6; Control mean = 9.8±6.8; group difference: t(36) = 2.23, p = 0.032].

When assessing participants’ understanding of the task instructions, 5 ASD participants offered additional anecdotal insight into their social distancing abnormalities, either by describing real-life events related to personal space violations (2 subjects), by providing somewhat atypical explanations for their behavior (2 subjects) or by demonstrating real-world abnormalities (1 subject). For instance, one participant described a recent event where he was explicitly told that he was standing inappropriately close to someone. Other subjects described that their discomfort was strictly due to sensory issues and restrictions (e.g., too much in my vision; can’t read body language when that close). Another participant demonstrated repeated personal space violations throughout his visit to the laboratory (e.g., touching the experimenter’s stomach, grabbing the experimenter’s hand, touching the experimenter’s face with both hands, etc.).

## Discussion

In Study 1, we found that social distancing differs between individuals with an ASD and their unaffected siblings, as assessed using parent-report SRS scores in a large sample comprised of 1532 individuals. ASD individuals were rated as being less aware of their closeness to others or of invading someone’s space compared to their unaffected siblings. This was true for 78.6% of ASD-sibling pairs, while the reverse was true for only 6.5% of pairs, demonstrating the robustness of this difference. Further, group differences in social distancing persisted across a wide range of ages (from 4 years to 18 years), as well as across the various ASD diagnostic sub-categories (i.e., Autistic Disorder, Asperger’s, and PDD-NOS). We also found that scores on the social and communication subscales of the ADI-R correlate positively with parent ratings of social distancing abnormality. Given that social distance is a socio-communicative signal, it makes sense that a relationship would be found for both of these domains of functioning (and not with the restricted and stereotyped behaviors subscale).

In Study 2, we further explored the nature and extent of social distancing abnormalities in a sample of high-functioning adults with autism, and in a more detailed way than which was possible based on the questionnaire data. Using a controlled experimental task, we demonstrated that the tight relationship we observed in the control group between personal space and interpersonal distance was disrupted in ASD (**Figure 4**). Additional evidence for social distancing abnormality comes from anecdotal reports and direct observation of violations of social distancing conventions by our participants, and from abnormal explanations for why particular distances are preferred (i.e., sensory explanations), demonstrating that these social distancing abnormalities can persist into adulthood. Furthermore, we documented the complete absence of a sense of personal space in 3 out of 18 participants ASD participants (17%), something not seen in any of the 20 control participants.

It is particularly noteworthy that abnormalities in aspects of social distancing in ASD were detected across these two experiments (Study 1 and Study 2), since they used very different methods and 2 very different populations of participants. Given the different methodologies, a direct comparison cannot be made between children/adolescents and older adults with ASD. However, some conclusions about whether social distancing abnormalities are present and how they manifest over development can still be drawn. In Study 1, we found that abnormalities in ASD are present early in life (i.e., present at 4 years of age, which was the earliest age assessed here), and while they diminish across age (Figure 3), they continue to be present and significantly abnormal into late adolescence/young adulthood (i.e., 18 years). Study 2 demonstrated that these abnormalities are still detectable well into adulthood in some individuals. At the group level, a more subtle abnormality was detected in the relationship between personal space and interpersonal distance, suggesting either a different mechanism by which social distancing skills had been acquired over development, or a different way in which social distancing decisions are made (e.g., less reliant on personal space/feelings of discomfort). Taken together, these studies demonstrate that social distancing abnormalities are widespread in childhood and adolescence, and may be a persistent, life-long feature of ASD, especially apparent in some individuals with an ASD.

In Study 1, scores on the parent-report measure of social distancing competency were most strongly correlated with several other items that also relate to social distancing. Two of these items were *a priori* items of interest (“Touches others in an unusual way…” and “walks in between two people who are talking”) since they explicitly assess violations of two aspects of social distancing - namely, personal space and social space. A third item, which actually had the highest correlation with item 55, is less obviously related to social distancing (“Knows when he or she is talking too loud or making too much noise”). However, one’s sense of space is a multimodal construct and can be violated by a number of sensory modalities [4], [20], including audition (e.g., talking too loud in a public area). Thus, it is not surprising that an individual that violates the space of another person tends to do so through more than one sensory modality.

In regard to the finding of a group difference in social distancing competency between individuals with an ASD and their unaffected siblings in Study 1, one potential concern is that families were preselected according to specific criteria that could have biased the results toward finding such a difference. For instance, inclusion of a family into the SSC dataset requires that there be only 1 affected individual, and that siblings are not diagnosed with or referred for possible ASD, along with additional exclusionary criteria applied to siblings (adaptive functioning levels below 70, identified as having a developmental delay other than Down Syndrome, diagnosed with schizophrenia or psychiatric disorders requiring treatment with more than 1 psychotropic medication, or having an Individualized Education Plan). The criteria for inclusion into the AGRE dataset, however, are less restrictive with regard to siblings, and allowed for inclusion of siblings that might have been referred for a possible ASD. Even within this AGRE sample, the group difference was still significant, the magnitude of this difference was larger compared to the SSC sample, and it remained significant even when we included those siblings that had elevated total SRS scores (indicative of clinically significant social impairment and a possible undiagnosed ASD). It is also worth pointing out that this concern regarding sibling selection would not influence the description of the social distancing phenotype within the ASD group (e.g., clinical correlates).

One particularly interesting finding, underscored by the integration of Study 1 and Study 2, is that social distancing abnormalities in ASD cannot be entirely explained by adaptive functioning (as measured with the Vineland) or intelligence. In Study 1, although there was a relationship between composite Vineland scores and social distancing in ASD (r = −0.19), this relationship alone could not account for the group difference in social distancing, since this difference persisted even when groups were carefully matched on composite Vineland scores (or specifically matched on the Vineland socialization domain). Similarly, in Study 2, an altered relationship between interpersonal distance preference and personal space was found in Study 2, where full-scale IQ scores were in the average to above average range (93–133). In fact, the three ASD participants without a sense of personal space had full-scale IQ scores of 100, 106 and 108. These findings together suggest that social distancing is a social competency that is at least partly separable from more general impairments in social, communicative, and daily living abilities as well as intelligence. We suggest that social distancing should be thought of as one specific facet of the composite set of abilities that constitute social functioning in real life; future studies should investigate the possibility that it may depend on partly dissociable underlying neurobiological mechanisms and/or genetic causes that could provide a window into subtypes of ASD.

Preliminary evidence regarding the neural systems underlying social distance regulation comes from a recent study that identified a critical role for the amygdala [21], a brain region with known anatomical and functional abnormalities in autism [22]. By studying a patient with complete bilateral lesions of the amygdala, Kennedy et al. [21] found that an intact amygdala is necessary for feelings of discomfort following personal space violations, thus helping to automatically regulate interpersonal distance. Furthermore, this prior study found that in neurotypical individuals, the amygdala exhibits greater activity when another person is standing close-by compared to when that person is far away. Given findings of anatomical abnormality [23]–[25] and functional abnormality [26] of the amygdala in individuals with ASD, it is possible that dysregulation of the relationship between personal space and interpersonal distance relates directly to amygdala dysfunction. The future demonstration of such a relationship could provide evidence that social distance regulation serves as an endophenotype for amygdala dysfunction in ASD.

Some limitations of the current studies should be noted. First, because the datasets analyzed in Study 1 were based on already acquired SRS data, our analysis was necessarily restricted to and limited by the specific items that comprise the SRS (and other phenotypic data). Given that these measures were not designed specifically to assess social distancing, we lacked the richness of measurement that one might obtain in an observational or experimental study. Another limitation is that, given the wording of item 55, we were only able to assess social distance violations arising from abnormally close proximity, and not social distance violations arising from abnormally far proximity. While our data clearly show that people with ASD generally are abnormal with respect to being too close, it remains an open question whether a subset of individuals with ASD might also sometimes be abnormally too far away from others. The wording of item 55 also inquires specifically about the child’s *knowledge* about social distancing, rather than the child’s behavior. Had the questionnaire explicitly assessed behavior, one might expect an even greater group difference, since rating a behavior is more objective and less open to interpretation and justification. The present study was unable to determine which specific factors may (or may not) influence social distancing in ASD. Past research in children with an ASD has shown that social distance is dependent on several factors, including the age and familiarity of the other person [8], opening the possibility that social distancing abnormalities in ASD may be highly context dependent, and that there may be at least some preserved aspects of social distance regulation, depending on the circumstances. Therefore, it should be emphasized that this study does not replace the need for observational and experimental research. Study 2 helped to address some of the above concerns by carrying out experimental laboratory tasks aimed at investigating the nature of social distancing abnormalities in more detail. However, this experiment also had limitations, especially given that the task was somewhat unnatural, especially in terms of the explicit nature of the task. It was made clear to participants that social distancing was being measured (both through instructions and also because of repeated measurements of distances), which is very different than typical social interactions where social distancing judgments are generally made in a more automatic and spontaneous manner. Thus, it is possible the explicit nature of the task may have masked real-world impairment that may still be present in some adults with ASD. This may be an additional factor underlying why our finding of a lack of an overall group difference in interpersonal distance preference in Study 2 was different from some previous reports (e.g., [13]). Other factors, including heterogeneity in symptom expression across individuals or social learning and adaptation over a protracted developmental timecourse may have also accounted for our lack of group-level differences in personal space and interpersonal distance measures.

From the current data, we are unable to determine the precise psychological mechanisms underlying social distancing abnormality in ASD. It is presently unclear whether abnormality in some individuals arises specifically from a lack of one’s own sense of personal space (which is observed in several participants in Study 2), from a lack of awareness of others’ personal space, a combination of the two, or abnormality in the mapping between one’s sense of personal space and interpersonal distance preference. This information would be crucial to know in order to develop strategic interventions [5], as each mechanism would dictate a different interventional emphasis (e.g., a focus on one’s own space, or a focus on other people’s personal space). However, the results from Study 2 might provide initial clues regarding one possible mechanism underlying social distancing abnormalities in ASD. Given the tight relationship between personal space and interpersonal distance in our control group, we suggest that decisions regarding interpersonal distance may normally be related to the feelings of discomfort – in other words, the larger one’s requirement for personal space, the proportionally greater interpersonal distance required by that individual. If feelings of discomfort were lacking or abnormal in individuals with ASD, then establishing a proper interpersonal distance would need to rely on other, non-visceral cues. While very preliminary, this hypothesis is supported by reports from two of our ASD participants, who described using sensory feedback, rather than visceral feelings of discomfort, to regulate their distance. Subsequent studies using a larger sample size, more sensitive and naturalistic measures of personal space and interpersonal distancing, and further probing how social distancing decisions are made by individuals with an ASD might help to provide further insight into these issues. In addition, further research aimed at understanding how personal space and interpersonal distance relate to and influence each other in both neurotypical subjects and those with ASD would be useful in this regard.

In sum, we have shown that social distance abnormalities are remarkably prevalent in ASD, and have detailed the relationships between social distancing and age, diagnosis, and clinical measures of social, communicative, and adaptive functioning. Using parent questionnaire data, in addition to interactive laboratory experiments and anecdotal report and observation, we have demonstrated that social distancing abnormalities persist over a wide range of ages and levels of functioning, and are still present in at least some cognitively-able high functioning adults with ASD. What we have not quantified here, however, is how abnormal regulation of social distance might negatively impact an individual’s real-world functioning in terms of the potentially serious consequences that might ensue. We have heard reports by parents of significant social and legal problems arising from personal space violations. Given the present findings, we suspect that this might be a widespread problem for individuals with an ASD and their families, and one that deserves careful consideration. Further understanding of this important aspect of social behavior, along with the psychological and neural mechanisms underlying its regulation and dysregulation, will be important in developing effective interventions aimed at ameliorating social distancing abnormalities, and potentially for improving social functioning in ASD more generally.
